This article has been retracted.

# Effect of Early Nutritional Assessment and Nutritional Support on Immune Function and Clinical Prognosis of Critically Ill Children

**DOI:** 10.1155/2022/7100238

**Published:** 2022-01-07

**Authors:** Jie Guo, Zixuan Jin, Yibing Cheng, Jun Su, Zheng Li, Zhipeng Jin

**Affiliations:** ^1^PICU, Children's Hospital Affiliated to Zhengzhou University (Henan Children's Hospital), Zhengzhou 450018, Henan, China; ^2^Xinhua Hospital of Shanghai Jiao Tong University, Shanghai 200092, China; ^3^PICU, Beijing Children's Hospital, Beijing 100000, China

## Abstract

The aim of this study was to study the effect of early nutritional assessment and nutritional support on immune function and clinical prognosis of critically ill children. 90 critically ill children at the same level of severity admitted to the pediatric intensive care unit (PICU) of our hospital (June 2019–June 2020) were chosen as the research objects and were equally separated into the experimental group and the control group by the random number table method. The children in the control group were admitted to the PICU according to the routine process, and the nutritional support was provided to the malnourished ones. After admission to the PICU, the children in the experimental group were given nutritional assessment, nutritional risk screening, and nutritional support according to the screening results. The PICU stay time and total hospitalization time of the experimental group were obviously shorter than those of the control group (*P* < 0.05), the hospitalization expenses of the experimental group were obviously lower than those of the control group (*P* < 0.05), the clinical outcomes and immune function of the experimental group were obviously better than those of the control group (*P* < 0.05), and the nutrition indicators of the experimental group were obviously higher than those of the control group (*P* < 0.05). Early nutritional assessment and nutritional support can effectively improve the immune function and reduce the incidence of adverse clinical outcomes of critically ill children, which are worthy of clinical application and promotion.

## 1. Introduction

Nutrition is essential for children's basal metabolism and growth, while malnutrition can hinder their growth and development. Malnutrition in critically ill children increases the incidence of infectious complications, leading to slow recovery, longer hospitalization time, and heavier mental and economic burden for their families. Children's energy reserves are lower compared with adults, but their growth and development need higher nutrition. In addition, some critically ill children fail to take in enough nutrients due to the poor dietary environment, leading to malnutrition [1–4]. The critically ill children are in sickness, and they have higher catabolism. If they fail to take in sufficient nutrients during hospitalization, it will lead to malnutrition or aggravated malnutrition. Moreover, chronic diseases and complications are common in critically ill children, so their incidence of malnutrition is higher. Thus, nutritional intervention is necessary for critically ill children. Nutritional intervention is mainly divided into nutritional risk screening, nutritional status assessment, and nutritional treatment. Rational nutritional support can effectively improve the nutritional status, reduce the incidence of complications, improve prognosis, and shorten the hospitalization time [5–7]. This study analyzed the effect of early nutritional assessment and nutritional support on immune function and clinical prognosis in critically ill children. In conclusion, early nutritional assessment and nutritional support for critically ill children can improve the immune function and the prognosis, shorten the hospitalization time, and relieve the economic burden and mental pressure of their families. The report is as follows.

## 2. Materials and Methods

### 2.1. General Data

90 critically ill children at the same level of severity admitted to the pediatric intensive care unit (PICU) of our hospital (June 2019-June 2020) were chosen as the research objects and were equally separated into the experimental group and the control group by the random number table method.

### 2.2. Inclusion Criteria

(1) All children met the diagnostic criteria of critical illness (met one of the criteria). (2) The children's clinical medical records were complete. (3) This study was approved by the hospital ethics committee. The children and their families were informed of the purpose and process of this study and signed the informed consent.

### 2.3. Exclusion Criteria

(1) The children who were unable to cooperate with the researchers. (2) The children with overnutrition. (3) The children who had received parenteral nutrition support in the past 3 months.

### 2.4. Methods

According to the routine admission process, the critically ill children in the control group were sent into the PICU. Their malnutrition was reported to the doctors, and then, nutritional support was provided to them according to the doctor's instructions.

After the critically ill children in the experimental group entered the PICU, the STRONGkids scale was used to screen their nutritional risks, and the subjective and comprehensive evaluation was carried out. It was observed that whether the children's muscle and subcutaneous fat were reduced, whether they had symptoms such as vomiting and excessive diarrhea, whether they reduced the diet and received the nutritional intervention of healthy diet before admission, whether they had severe pain that prevented them from eating, and whether they had experienced weight loss and slow growth in recent months. The children were also checked for anorexia nervosa, chronic heart diseases, enteritis, abdominal diseases, burns, and expected major surgeries. The children's nutritional status was evaluated, and doctors needed to work with nutritionists to develop nutritional intervention plans for them. The children's nutritional status should be reevaluated every week, and then, the nutritional support route and dosage would be adjusted by the doctors and nutritionists according to the actual situation [8, 9].

### 2.5. Observation Indexes

The clinical indexes of the two groups were recorded and compared, including the PICU stay time, total hospitalization time, and total hospitalization expenses.

The clinical outcomes of the two groups were compared.

Before and after the intervention, 5 ml of peripheral blood of the two groups was collected, and the serum was centrifuged to monitor immunological indexes. The levels of C3, C4, IgA, IgM, and IgG were detected by enzyme-linked immunosorbent assay. The instructions were strictly followed to perform the abovementioned steps.

The levels of albumin, prealbumin, and hemoglobin of the two groups were detected by using an automatic biochemical analyzer, and the nutrition indicators of the two groups were compared.

### 2.6. Statistical Treatment

The data processing software selected in this study was SPSS20.0, and the selected drawing software was GraphPad Prism 7 (GraphPad Software, San Diego, USA). This study included count data and measurement data, using the *x*^2^ test, *t*-test, and normality test methods. When *P* < 0.05, the difference was statistically significant.

## 3. Results

### 3.1. Comparison of the General Data

No significant difference in age, BMI, gender, and residence was found between the two groups (*P* > 0.05), indicating comparability, see Table 1.

### 3.2. Comparison of the Clinical Indexes

The clinical indexes of the experimental group were lower than those of the control group (*P* < 0.05), see Table 2.

### 3.3. Comparison of the Clinical Outcomes

The clinical outcomes of the experimental group were obviously better than those of the control group (*P* < 0.05), see Table 3.

### 3.4. Comparison of the Immunological Indexes

#### 3.4.1. Comparison of the IgA Levels

After intervention, the IgA level in the experimental group was obviously lower than that in the control group (*P* < 0.05), see Figure 1.

#### 3.4.2. Comparison of IgM Levels

After intervention, the IgM level in the experimental group was obviously lower than that in the control group (*P* < 0.05), see Figure 2.

#### 3.4.3. Comparison of the IgG Levels

After intervention, the IgG level in the experimental group was obviously lower than that in the control group (*P* < 0.05), see Figure 3.

#### 3.4.4. Comparison of the C3 Levels

After intervention, the C3 level in the experimental group was obviously lower than that in the control group (*P* < 0.05), see Figure 4.

#### 3.4.5. Comparison of the C4 Levels

After intervention, the C4 level in the experimental group was obviously lower than that in the control group (*P* < 0.05), see Figure 5.

### 3.5. Comparison of the Nutrition Indicators

The nutrition indicators of the experimental group were obviously higher than those of the control group (*P* < 0.05), see Table 4.

## 4. Discussion

At present, sufficient attention has not been paid to the nutritional treatment of critically ill children in clinical practice and the nutritional treatment is not standardized. The children's nutritional risks have not been screened in time. Thus, the malnutrition of critically ill children is neglected [10–13]. Due to the insufficient awareness of adverse clinical outcomes caused by malnutrition of children and the lack of knowledge about nutritional treatment, standardized nutritional treatment is not available. The critically ill children are in a serious condition, some of whom suffer from congenital diseases, inherited metabolic diseases, and chronic diseases, leading to chronic malnutrition. If nutritional intervention is not given to the children in time, it will aggravate the malnutrition and directly affect their clinical outcomes [14–16]. The critically ill children with malnutrition generally lack micronutrients such as iron, zinc, and vitamin. The level of immune cell factors is affected by the levels of micronutrients and auxiliary factors. Children lacking micronutrients have a decline in immune function and are highly prone to infection. In severe cases, their immune function may be defective. Therefore, the level of micronutrients is important in the process of nutritional support for critically ill children, and micronutrients should be appropriately provided to improve their nutritional status. For critically ill children who are in the recovery and stability period and have normal gastrointestinal tract function, oral intake is allowed, but the type and amount of diet need to be controlled [17–20]. Food is provided according to the children's preferences to improve their interest in eating and increase their intake of energy and protein. It can also avoid wasting food and save food costs. Some critically ill children need to be treated with mechanical ventilation, and the mechanical ventilation time will be prolonged due to the respiratory muscle weakness caused by insufficient nutritional support. Mechanical ventilation has a direct impact on the energy intake of children and leads to their poorer nutritional status, and the insufficient intake of energy prolongs the mechanical ventilation time, thus forming a vicious circle [21–24]. This study showed that the immune function of the experimental group was obviously better than that of the control group (*P* < 0.05), which was consistent with the research results of Jonckheer et al. [25]. Their paper showed that the immunological indexes C3, C4, IgA, IgM, and IgG in the experimental group were (0.37 ± 0.34) *μ*mol/L, (0.14 ± 0.12) *μ*mol/L, (2.03 ± 0.92) *μ*mol/L, (0.87 ± 0.45) *μ*mol/L, and (5.52 ± 1.68) *μ*mol/L, respectively, while those in the control group were (0.77 ± 0.35) *μ*mol/L, (0.56 ± 0.08) *μ*mol/L, (2.95 ± 0.89) *μ*mol/L, (1.28 ± 0.54) *μ*mol/L, and (7.55 ± 1.82) *μ*mol/L, respectively.

## 5. Conclusions

The immune function in the experimental group was obviously better than that in the control group (*P* < 0.05), indicating that nutritional support for critically ill children could improve their immune function, promote their recovery, and improve their clinical outcomes.

In conclusion, early nutritional assessment and nutritional support for critically ill children can improve the immune function and the prognosis, shorten the hospitalization time, and relieve the economic burden and mental pressure of their families. Therefore, they are worthy of clinical application and promotion.

## Figures and Tables

**Figure 1:** Comparison of IgA levels ($\bar{X}\pm s$). The horizontal axis from left to right represents before intervention and after intervention, and the vertical axis represents the IgA level (*μ*mol/L). In the experimental group, the IgA levels before and after intervention were (4.79 ± 0.93) *μ*mol/L and (2.02 ± 0.91) *μ*mol/L, respectively. In the control group, the IgA levels before and after intervention were (4.83 ± 0.89) *μ*mol/L and (2.94 ± 0.88) *μ*mol/L, respectively. ^*∗*^The IgA levels of the experimental group before and after intervention were obviously different (*t* = 21.807, *P* < 0.001). ^*∗∗*^The IgA levels of the control group before and after intervention were obviously different (*t* = 16.070, *P* < 0.001). ^*∗∗∗*^The IgA levels of the two groups after intervention were obviously different (*t* = 9.886, *P* < 0.001).

**Figure 2:** Comparison of IgM levels ($\bar{X}\pm s$). The horizontal axis from left to right represents before intervention and after intervention, and the vertical axis represents the IgM level (*μ*mol/L). In the experimental group, the IgM levels before and after intervention were (1.86 ± 0.76) *μ*mol/L and (0.86 ± 0.44) *μ*mol/L, respectively. In the control group, the IgM levels before and after intervention were (1.87 ± 0.74) *μ*mol/L and (1.27 ± 0.53) *μ*mol/L, respectively. ^*∗*^The IgM levels of the experimental group before and after intervention were obviously different (*t* = 7.639, *P* < 0.001). ^*∗∗*^The IgM levels of the control group before and after intervention were obviously different (*t* = 4.422, *P* < 0.001). ^*∗∗∗*^The IgM levels of the two groups after intervention were obviously different (*t* = 3.993, *P* < 0.001).

**Figure 3:** Comparison of IgG levels ($\bar{X}\pm s$). The horizontal axis from left to right represents before intervention and after intervention, and the vertical axis represents the IgG level (*μ*mol/L). In the experimental group, the IgG levels before and after intervention were (12.49 ± 4.36) *μ*mol/L and (5.51 ± 1.69) *μ*mol/L, respectively. In the control group, the IgG levels before and after intervention were (12.47 ± 4.33) *μ*mol/L and (7.54 ± 1.81) *μ*mol/L, respectively. ^*∗*^The IgG levels of the experimental group before and after intervention were obviously different (*t* = 10.013, *P* < 0.001). ^*∗∗*^The IgG levels of the control group before and after intervention were obviously different (*t* = 7.047, *P* < 0.001). ^*∗∗∗*^The IgG levels of the two groups after intervention were obviously different (*t* = 5.499, *P* < 0.001).

**Figure 4:** Comparison of C3 levels ($\bar{X}\pm s$). The horizontal axis from left to right represents before intervention and after intervention, and the vertical axis represents the C3 level (*μ*mol/L). In the experimental group, the C3 levels before and after intervention were (1.55 ± 0.47) *μ*mol/L and (0.39 ± 0.36) *μ*mol/L, respectively. In the control group, the C3 levels before and after intervention were (1.52 ± 0.46) *μ*mol/L and (0.76 ± 0.34) *μ*mol/L respectively. ^*∗*^The C3 levels of the experimental group before and after intervention were obviously different (*t* = 13.484, *P* < 0.001). ^*∗∗*^The C3 levels of the control group before and after intervention were obviously different (*t* = 8.913, *P* < 0.001). ^*∗∗∗*^The C3 levels of the two groups after intervention were obviously different (*t* = 5.419, *P* < 0.001).

**Figure 5:** Comparison of C4 levels ($\bar{X}\pm s$). The horizontal axis from left to right represents before intervention and after intervention, and the vertical axis represents the C4 level (*μ*mol/L). In the experimental group, the C4 levels before and after intervention were (1.02 ± 0.34) *μ*mol/L and (0.13 ± 0.11) *μ*mol/L, respectively. In the control group, the C4 levels before and after intervention were (1.04 ± 0.31) *μ*mol/L and (0.55 ± 0.09) *μ*mol/L, respectively. ^*∗*^The C4 levels of the experimental group before and after intervention were obviously different (*t* = 16.707, *P* < 0.001). ^*∗∗*^The C4 levels of the control group before and after intervention were obviously different (*t* = 10.183, *P* < 0.001). ^*∗∗∗*^The C4 levels of the two groups after intervention were obviously different (*t* = 19.823, *P* < 0.001).

**Table 1:** Comparison of general data (*n* (%)).

	Experimental group (*n* = 45)	Control group (*n* = 45)	*X* ^2^ or *t*	*P*
Age (years)			0.279	0.781
	3.12 ± 0.53	3.15 ± 0.49		
BMI (kg/m^2^)			0.387	0.699
	11.23 ± 0.32	11.26 ± 0.41		
Gender			0.180	0.671
Male	26 (57.78)	24 (53.33)		
Female	19 (42.22)	21 (46.67)		
Residence			0.182	0.670
Cities and towns	27 (60.00)	25 (55.56)		
Countryside	18 (40.00)	20 (44.44)		

**Table 2:** Comparison of clinical indexes ($\bar{X}\pm s$).

Items	*n*	PICU stay time/d	Total hospitalization time/d	Total hospitalization expenses/ten thousand Yuan
Experimental group	45	7.49 ± 2.31	14.37 ± 4.28	3.41 ± 1.12
Control group	45	9.69 ± 2.37	17.41 ± 4.21	3.92 ± 1.21
*t*		4.459	3.397	2.075
*P*		<0.001	0.001	0.041

**Table 3:** Comparison of clinical outcomes (*n* (%)).

Items	*n*	Recovery	Improvement	Giving up treatment	Death
Experimental group	45	24 (53.33)	17 (37.78)	3 (6.67)	1 (2.22)
Control group	45	17 (37.78)	19 (42.22)	2 (4.44)	7 (15.56)
*X* ^2^		2.195	0.185	0.212	4.939
*P*		0.138	0.667	0.645	0.026

**Table 4:** Comparison of nutrition indicators ($\bar{X}\pm s$).

Items	*n*	Albumin		Prealbumin		Hemoglobin	
		Before intervention	After intervention	Before intervention	After intervention	Before intervention	After intervention
Experimental group	45	32.34 ± 1.47	39.87 ± 3.96	26.54 ± 2.37	36.57 ± 4.89	112.54 ± 2.76	131.47 ± 3.54
Control group	45	32.54 ± 2.03	34.74 ± 3.74	26.61 ± 2.29	31.34 ± 5.13	112.61 ± 3.04	118.42 ± 6.07
*T*		0.535	6.318	0.142	4.590	0.114	12.458
*P*		>0.05	>0.05	>0.05	<0.05	>0.05	<0.05

## Data Availability

The datasets used and/or analyzed during the current study are available from the corresponding author on reasonable request.
